# A Data Collection Method for Mobile Wireless Sensor Networks Based on Improved Dragonfly Algorithm

**DOI:** 10.1155/2022/4735687

**Published:** 2022-05-17

**Authors:** Yinggao Yue, Dongwan Lu, Yong Zhang, Minghai Xu, Zhongyi Hu, Bo Li, Shuxin Wang, Haihua Ding

**Affiliations:** ^1^School of Intelligent Manufacturing and Electronic Engineering, Wenzhou University of Technology, Wenzhou, 325035, China; ^2^Intelligent Information Systems Institute, Wenzhou University, Wenzhou, 325035, China; ^3^Computer School, Hubei University of Arts and Science, Xiangyang, 441053, China; ^4^Key Laboratory of Intelligent Image Processing and Analysis, Wenzhou, China; ^5^Wenzhou Key Laboratory of Intelligent Lifeline Protection and Emergency Technology for Resilient City, Wenzhou University of Technology, Wenzhou, 325035, China

## Abstract

For the sensing layer of the Internet of Things, the mobile wireless sensor network has problems such as limited energy of the sensor nodes, unbalanced energy consumption, unreliability, and long transmission delay in the data collection process. It is proved by mathematical derivation and theory that this is a typical multiobjective optimization problem. In this paper, the optimization goal is to minimize the energy consumption and improve the reliability under time-delay constraints and propose a path optimization mechanism to optimize the mobile Sink of mobile wireless sensor networks based on the improved dragonfly optimization algorithm. The algorithm takes full advantage of the abundant storage space, sufficient energy, and strong computing power of the mobile Sink to ensure network connectivity and improve network communication efficiency. Through simulation comparison and analysis, compared with random movement method, artificial bee colony algorithm, and basic dragonfly optimization algorithm, the energy consumption of the network is reduced, the lifespan of the network is increased, and the connectivity and transmission delay of the network are improved. The proposed algorithm balances the energy consumption of the sensors nodes to meet the network service quality and improve the reliability of the network.

## 1. Introduction

In recent years, the Internet of Things technology has received the attention and in-depth development of a wide range of researchers and has been rapidly applied in fields such as smart logistics, smart factories, robots, Industry 5.0, smart medical care, and smart industry and agriculture [1]. The data perception collection technology of the wireless sensor network at the perception layer of the Internet of Things is the key technology at the bottom of the realization of various functions of the Internet of Things and has been widely valued by experts and scholars. Data collection is an important stage of the application of wireless sensor networks [2]. In multihop communication, because nodes close to the Sink undertake more data forwarding tasks, their energy consumption is faster, and energy holes are easily formed. Once an energy hole appears, the network is divided. Therefore, balancing the energy consumption between nodes is the key to avoiding energy holes [3].

Due to random deployment, complex environments, and limited node resources, single-path routing data transmission methods are likely to cause imbalance in network energy consumption. The use of mobile Sink for data collection can greatly reduce the multihop transmission of data and at the same time shorten the transmission distance between the node and the mobile Sink, save the energy consumption of the sensor node, and improve the reliability of the network [4]. In order to maximize the amount of data collection, mobile Sink data collection strategies are often used. However, due to the slow moving speed of the mobile Sink, the use of the mobile Sink will increase the data transmission delay. Therefore, optimizing the data transmission delay is the key to the mobile strategy based on the Sink [5].

The path optimization design of mobile Sink not only considers the length of the data transmission path but also considers issues such as energy saving and network energy balance. Considering the trade-off between energy consumption, reliability, and delay [6], the path optimization of mobile wireless sensor networks is a typical multiobjective optimization problem. The movement of the Sink node can effectively balance the network energy consumption, and planning the path of the mobile Sink is the key to this strategy [7]. The simplest method is to traverse each node and then directly receive the sensing data. But this method does not solve the traveling salesman problem (TSP). The TSP is how to traverse all nodes in the shortest path. However, as the network scale increases, the number of nodes increases sharply, and it is no small challenge to get the shortest path [3].

Aiming at the above problems, the optimization goal is reduced to minimize the energy consumption and improve the reliability under time-delay constraints, and an improved dragonfly algorithm is proposed to optimize the movement path of the mobile Sink. The proposed algorithm constructs a highly invulnerable network topology, reduces the length of data transmission links, balances energy consumption, and ensures the robustness and availability of wireless sensor networks at the perception layer of the Internet of Things. In this work, a data collection strategy for wireless sensor networks based on energy efficiency and collaborative optimization is proposed. In comparison with the current general selection approaches, the main contributions of our work in this paper can be summarized as follows:

1. Characterize the issues of the data collection for WSNs, and classify the current data collection of WSNs
2. The data collection problem of mobile Sink for WSNs is compared with the traveling salesman problem, and an energy-saving and efficient data collection method of WSNs based on the improved dragonfly algorithm (IDA) is proposed
3. Evaluate the performance of the proposed algorithms by comparing them with the data collection methods of the random walk, artificial bee colony (ABC) algorithm, and dragonfly algorithm (DA)

## 2. Related Work

Reliable and efficient data collection is a key issue in the application of wireless sensor networks. The current research on data collection methods of wireless sensor networks is mainly in the two following aspects: static sensor network data collection and mobile sensor network data collection. The research of this paper is mainly in the data collection research of mobile wireless sensor network [8].

*Data Collection Algorithm Based on Static Wireless Sensor Network*. In traditional static WSNs, once the sensor nodes are deployed, they generally remain stationary. After the sensor node is started, it will start a process of detecting other sensor nodes around it. After a period of time, the network topology is formed and the sensor node starts to work. They transmit the data they detect from various directions in a multihop transmission mode to a node capable of complex data processing and calculation. Alrashidi et al. [9] proposed an advanced cluster concept for energy efficiency clustering and data collection in industrial WSNs, in order to improve the network's lifetime and minimize power consumption. The remaining energy, the degree of connectivity, and the distance between the cluster head node and other nodes are comprehensively considered. At the same time, a routing method based on artificial intelligence is also proposed to solve the problem of data collection. Liu and Chen [10] constructed a data collection tree for the WSNs data collection problem and proposed an algorithm for maximizing the sampling rate of sensor nodes during the network operation stage. The results show that the method is effective and robust in data collection. Soleymani et al. [11] used the symmetrical correlation of sensor data to reduce the energy consumption of sensor nodes and proposed a data collection method based on decision trees, autoregressive integrated moving averages, and Kalman filtering methods. This method effectively increases the life of the network and reduces the energy consumption of the network. Li et al. [12] proposed a data acquisition scheme based on the denoising autoencoder to solve the problem that the result of sparse transformation of sensor data is not necessarily the sparsest. The proposed scheme has higher data compression rate, lower energy consumption, more accurate data reconstruction, and faster data reconstruction speed.

Generally speaking, the process from the generating node of the data packet to the final receiving node of the data packet is often accompanied by the forwarding of a large number of data packets. All sensor nodes located on the forwarding path will consume twice as much energy. What is more serious is the fact that the closer the sensor node to the final receiving node of the data packet, the faster the energy consumption. It is conceivable that the use of this method of data collection has many negative effects on the performance of the network. Liu et al. [13] proposed an iterative data association and trajectory planning data collection strategy for the optimization of network energy consumption for optimal data collection, which effectively improved the efficiency of data collection. Cohen et al. [14] proposed a data collection protocol based on the principle of information theory to match the physical layer, access control, and traffic patterns. At the same time, it also provides a simple data encoding structure and corresponding encoding and decoding procedures, which greatly improves the efficiency of data collection. Miao et al. [15] proposed a multihop weighted (MWR) algorithm to approximate the optimal solution for the goal of minimizing the data collection delay of WSNs. The results show that the proposed MWR algorithm effectively reduces the total data collection delay in different network scenarios and at the same time reduces the network energy consumption. Lu et al. [16] proposed a data collection mechanism for space-time correlation perception for event-driven sensor networks. On the Sink node, the sensed data is gathered based on the temporal and spatial correlation, and the particle swarm optimization algorithm is used to obtain the best data collection path. The results show that the proposed algorithm can effectively reduce the amount of data transmission and reduce network delay and energy consumption.

*Data Collection Scheme Based on Mobile Data Collector*. In order to interrupt the long data packet forwarding path, the idea of a mobile data collector has gradually come out. The mobile data collector is generally a robot or a small car with an antenna, which can roam the entire wireless sensor network. It starts from the data processing center, stops at a certain cluster head node, starts to collect the data retained in the surrounding sensor nodes within a certain range, then moves to the next cluster head node, and finally returns to the data processing center for data reporting. Ma et al. [17] studied the data collection of mobile wireless sensor networks (WSNs) assisted by multiple unmanned aerial vehicles (UAVs). Aiming at such a highly dynamic network, a balancing algorithm is proposed for collision-free communication between mobile nodes and multiple UAVs. The results show that the proposed algorithm has certain applicability in real scenes. Saranya et al. [18] proposed a novel energy-saving data collection scheme. The data collection of the mobile Sink is completed by a dynamic polling mechanism based on the arrival rate of cluster head nodes. The results show that the proposed algorithm is superior to LEACH algorithm and energy-aware multihop routing protocol (M-GEAR) in terms of lifetime, latency, and throughput. Kumar and Dash [19] considered the use of mobile Sinks to move along a prespecified path at a constant speed for data collection, as well as the use of network flow methods for effective data forwarding. The proposed scheme has significant effects in terms of total data collection and energy efficiency. Lin et al. [20] proposed a DDF data collection mechanism. In each round of cluster head selection and tree topology stage, mobile Sinks are used to collect data in heterogeneous WSNs (HWSNs). This method prolongs the lifetime of the network and improves the coverage of monitoring. Ang et al. [21] proposed an analysis method to determine the node energy consumption of the LS-WSNMDC scheme, using a mobile data collector (MDC) for data collection. At the same time, a model to determine the optimal number of clusters to minimize energy consumption is given. This method reduces network energy consumption and prolongs the lifetime of the network.

By reducing the number of communication hops, reducing the data packet loss rate, and constructing an optimal movement path, energy efficiency can be improved. However, how to plan the path based on the set of cluster head nodes and construct the optimal mobile Sink path planning is still a challenge. Roy et al. [22] proposed an efficient data collection protocol for wireless sensor networks through mobile data collectors focusing on service quality. Ant colony optimization is used to determine the best trajectory for accessing all data collection points. The results show the effectiveness of the proposed protocol in terms of network life, total energy consumption, end-to-end delay, and packet loss rate. Byun [23] planned the optimal path problem of the mobile Sink collector and proposed a cost-balancing algorithm based on the mobile Sink. This method can achieve data collection delay and energy consumption based on adaptive area division and dynamic polling point selection. The results verify the superiority of the proposed algorithm. Kaur and Grewal [24] proposed a mobile Sink data collection technology (PSODSM) based on particle swarm optimization (PSO) to reduce the energy consumption of WSNs and prolong the lifetime of the network. Roy et al. [25] found a balance between energy conservation and data transmission delay to ensure the data transmission hop of each cluster. Using ant colony optimization (ACO) algorithm to form the moving path of the mobile Sink, a near-optimal solution is proposed, which is more effective in terms of network life and energy consumption. Pang et al. [26] proposed a collaborative data collection scheme using multiple mobile Sink nodes, using a dynamic clustering algorithm to cluster randomly arranged sensor nodes. At the same time, a path-based equalization algorithm (PEABR) is proposed to adjust the path of the mobile Sink, and the result shows the feasibility and effectiveness of the algorithm. In order to overcome the limitations of traditional data collection methods in large-scale farmland wireless sensor networks, Yang et al. [27] introduced mobile Sink and proposed a path planning strategy for mobile Sink based on virtual potential field. The results show that the method has good transmission efficiency and prolongs the lifetime of the network. Considering the above issues, the researchers propose a one-stop framework solution for mobile data collection. Considering the parallel data upload, the framework in [23] solves the data upload delay very well, thereby greatly reducing energy consumption. Literature [25] considers the conflict between longer network survival time and shorter data delay as a whole. It considers the scheduling and interaction between WSN node layer, cluster head layer, and mobile data collector layer. Their results show that this framework-based solution can be applied to many scenarios and has a very good performance improvement.

In summary, in order to overcome the energy hole problem, reduce network energy consumption, and improve data collection efficiency, consider Sink node movement. The data collection of the mobile sensor node mainly involves the movement path selection of the Sink node and the energy consumption of data collection. Considering multiple factors, a data collection algorithm for a wireless sensor network with mobile Sink is proposed. Establish a data collection optimization model including constraints such as Sink movement path selection constraints, data flow constraints, energy consumption constraints, and link constraints. The optimized and improved dragonfly optimization algorithm is used to solve the optimization model and obtain the optimal solution. That is, the Sink node can find a better moving path, and the sensor node can find a better data transmission scheme, thereby improving the network's survival time and data transmission rate, reducing the length of the moving path and the average node energy consumption, and improving the reliability of the network.

## 3. Problem Description

In the clustered data collection process of mobile wireless sensor networks, we consider a data collection scenario in the case of a mobile Sink. In the clustering scene, the detected area is divided into layers. Divided into two layers, the bottom layer is mainly composed of ordinary sensor nodes, and the main job is to collect data. The upper layer is mainly composed of cluster head nodes. The task of the cluster head is to collect and distribute receipts. The cluster head assigns tasks to the member nodes in the cluster, and the member nodes in the cluster transfer the collected data to the cluster head. The cluster head first performs data fusion. When the Sink moves to the communication range of the cluster head, it is then forwarded to the mobile Sink.

In this paper, the data collection process of the mobile Sink is based on LEACH clustering. The cluster head will also change the clustering interval in real time according to the change in the number of data collection polls. The Sink node does not need to know the location of the common node during the data collection process and only receives the data forwarded by the cluster head node.

This article defines the following definitions for the mobile Sink movement path optimization problem in the mobile wireless sensor network at the perception layer of the Internet of Things.

**Definition 1 .**

The minimum energy consumption movement path. In the data collection process of the mobile wireless sensor network at the perception layer of the Internet of Things, in order to meet the constraints of time delay, energy consumption, and network reliability, this method enables the collected data to be transmitted from the cluster head node to the Sink node with the smallest total energy consumption and the shortest total path length.

**Definition 2 .**

The shortest path of movement. It is defined as the shortest moving path length for the mobile Sink to collect data from all cluster head nodes in the monitoring area.

Assume that the initial position of the mobile Sink for data collection during each polling work is *C0*. The moving speed of the mobile Sink is *V*_*Sink*_, and the total maximum time delay of data collection is *D*, so the maximum moving path length of the mobile Sink is *L* = *V*_*Sink*_ × *D*. Assuming that the parameters *J* and *Q* = (*q*_*i*_) are the cluster head node set and the corresponding number set, respectively, parameter *N* represents the total set of nodes that need to be migrated. According to the scene model described above, the total energy consumption of the mobile Sink for data collection in the monitoring area is

(1) $$\begin{array}{c} E_{\text{Total}}=\sum_{i=1}^{\lfloor N\rfloor }\left(2E_{\text{elec}}\times T_{i}+E_{i}^{p}\left(1\right)+E_{i}^{p}\left(2\right)+\cdots +E_{i}^{p}{\left(T_{i}\right)}_{q_{i}}+E_{\text{elec}}\times \sum_{i=1}^{\left|J\right|}q_{i}-2E_{\text{elec}}\sum_{i=1}^{\left|N_{0}\right|}q_{i}\right), \end{array}$$

(2) $$\begin{array}{c} \min\sum_{i=1}^{\lfloor N\rfloor }\left(2E_{\text{elec}}\times T_{i}+E_{i}^{p}\left(1\right)+E_{i}^{p}\left(2\right)+\cdots +E_{i}^{p}\left(T_{i}\right)q_{i}\right), \end{array}$$

(3) $$\begin{array}{c} \sum_{l\in V_{f}}y_{l}\leq K, \end{array}$$

(4) $$\begin{array}{c} \sum_{l\in V_{s}}x_{ik}\leq T\left|V_{s}\right|y_{k},\;k\in V_{f}, \end{array}$$

(5) $$\begin{array}{c} \text{s.t.}TSP\left(S_{v}\right)\leq L. \end{array}$$

The parameters are defined as follows: parameter *T*_*i*_ is the total number of hops when the Sink node moves to the nearby cluster head node with the minimum energy consumption and minimum distance. *E*_*i*_^*p*^(*m*) represents the network energy consumption in the current *m*-th hop situation, where *m*∈[1, *T*_*i*_], and parameter *N*_*0*_ represents the set of mobile Sinks that can be moved to the cluster head node. Parameter *TSP*(*S*_*v*_) represents the set of the sensor nodes to be visited by mobile Sink. Parameter *L* is the total distance traveled by the mobile Sink to collect all cluster head nodes in the monitoring area. Equation (1) is our optimization objective function, and equations (2)–(5) are constraints. Equation (1) expresses the energy required for the mobile Sink to collect all the data in the monitoring area once. Equation (2) indicates that the energy consumption of all cluster head nodes in the data collection process is minimized. Equation (3) expresses the shortest distance from the initial point where the mobile Sink collects the monitoring area data and returns to the initial point after the location of the visited cluster head node. This problem can be understood as the collection of the minimum path of all the cluster head nodes in the mobile Sink, which is similar to the problem of obtaining the shortest distance through the optimization of the traveling salesman. Constraint condition (4) is that the number of feasible positions searched by the mobile Sink is at most *K*. Constraint condition (5) guarantees that the mobile Sink can only send data within the communication range of the sensor node *x*_*i*_. The path optimization problem of the mobile Sink is to obtain the mobile Sink to ensure the minimum energy consumption, path optimization, and high reliability of the monitoring area for data collection. This is a combined optimization problem. In this paper, a mobile sensor network data collection method based on the improved dragonfly algorithm is proposed to improve the efficiency and reliability of data collection, prolong the lifetime of the network, and reduce the energy consumption of the network.

## 4. Improved Dragonfly Algorithm

### 4.1. Dragonfly Algorithm

Dragonfly algorithm (DA) was proposed by Australian scholar Seyedali Mirjalili. The design of dragonfly algorithm is inspired by the unique social behavior of dragonflies [28]. The algorithm mainly searches for the global optimal solution to the optimization problem by simulating the predation behavior of dragonflies [29]. According to the behavior of dragonflies in the predation process, there are five main social behaviors of dragonflies, namely, (1) collision avoidance behavior, to avoid collisions with neighboring individuals; (2) the grouping behavior that is consistent with the average speed of neighboring individuals; (3) gathering behavior, gathering to the center of neighboring individuals; (4) foraging behavior, close to the food source; and (5) the behavior of avoiding enemies and staying away from natural enemies [30]. Compared with other algorithms such as particle swarm optimization (PSO), artificial bee colony (ABC) algorithm, and gray wolf optimization (GWO) algorithm, dragonfly algorithm has broader application prospects in the fields of path optimization, fault diagnosis, and image processing [31–33].

The social behavior of dragonflies is divided into static behavior and dynamic behavior. In the static behavior, dragonflies usually forage in a certain range in the form of small groups, and their main behaviors are gathering, foraging, and avoiding enemies. In dynamic behavior, if a small group of dragonflies find food, they will notify other small groups to come. At this time, the main behaviors are collision avoidance, gathering, and formation.

In the process of function solving, static behavior corresponds to global optimization, and dynamic behavior corresponds to local development. The following is the mathematical description of the dragonfly algorithm. Initially generate *m* dragonfly populations in the *N*-dimensional space, and the position of the *i*-th (*i*=1,2,3,…, *m*) dragonfly in the population represents *X*_*i*_=(*X*_*i*1_, *X*_*i*2_, *X*_*i*3_,…*X*_*iN*_). The fitness function value *f*(*x*) corresponding to the dragonfly population is calculated and compared. At the same time, the position of the dragonfly with the largest current fitness value is selected as the food source position, and the position of the dragonfly with the smallest fitness value is selected as the position of the natural enemy, and then the current individual location is updated according to the five behaviors of the dragonfly.

The specific formula is as follows [34]:

(1) Collision avoidance behavior: avoid collisions between dragonflies and neighboring individuals.
  (6) $$\begin{array}{c} S_{i}=\sum_{j=1}^{W}\left(X-X_{j}\right), \end{array}$$
where parameter *X* is the position of the current dragonfly. Parameter *X*_*j*_ is the position of the *j*-th adjacent dragonfly. Parameter *W* is the number of neighboring dragonflies.
(2) Teaming behavior: the speed between adjacent individuals tends to be the same.
  (7) $$\begin{array}{c} A_{i}=\frac{\sum_{j=1}^{W}V_{j}}{W}, \end{array}$$
where parameter *V*_*j*_ is the speed of the *j*-th adjacent dragonfly.
(3) Congregation behavior: dragonflies tend to congregate towards the center of neighboring individuals.
  (8) $$\begin{array}{c} C_{i}=\frac{\sum_{j=1}^{W}X_{j}}{W}-X. \end{array}$$
(4) Foraging behavior: the it is the attraction of dragonflies to food.
  (9) $$\begin{array}{c} F_{i}=X^{+}-X, \end{array}$$
where parameter *X*^*+*^ is the location of the food source.
(5) Avoidance of enemies: it is the repulsive force of dragonflies against natural enemies.
  (10) $$\begin{array}{c} E_{i}=X^{-}+X, \end{array}$$
where parameter *X*^−^ is the location of the natural enemy.
In addition to the above five behaviors, in order to more accurately simulate the movement of the dragonfly, Mirjalili introduced two more quantities: the step vector (*dX*) and the position vector (*X*). The calculation formula of the step length vector is as follows (this is the step length defined dimension by dimension) [35]:
  (11) $$\begin{array}{c} \Delta X_{t+1}=\left(sS_{i}+\alpha A_{i}+cC_{i}+fF_{i}+eE_{i}\right)+\omega \Delta X_{i}, \end{array}$$
where parameter *s* represents the separation weight, *α* represents the team weight, *c* represents the aggregation weight, *f* represents the food factor, and *e* represents the natural enemy factor. Parameter *S*_*i*_ represents the position of the *i*-th individual after separation, and *A*_*i*_ represents the position of the *i*-th individual after forming a team. Parameter *C*_*i*_ represents the position of the *i*-th individual after gathering, *F*_*i*_ represents the position of the dragonfly food of the *i*-th individual, and *E*_*i*_ represents the position of the natural enemy of the *i*-th individual dragonfly. Parameter *w* represents the weight of inertia. Parameter *t* represents the current iteration number [36]. The location is updated as follows.
(6) If there are dragonfly individuals nearby, update as follows:
  (12) $$\begin{array}{c} X_{t+1}=X_{t}+\Delta X_{t+1}. \end{array}$$
(7) If there is no dragonfly nearby, perform Levi flight:
  (13) $$\begin{array}{c} X_{t+1}=X_{t}+\text{Levy}\left(d\right)\times X_{t}, \end{array}$$
where parameter *d* is the dimension of the problem to be solved.

### 4.2. Improved Dragonfly Algorithm

#### 4.2.1. Chaos Initialization

The population initialization plays a vital role in the solution accuracy and convergence speed of the DA. When the standard DA is initialized, a random initialization method is generally adopted to determine the position and moving step length of the dragonfly. The disadvantage is that the convergence speed will be affected when the dragonfly is far away from the food source. Chaotic motion has the characteristics of regularity, randomness, and ergodicity. This process is not convergent but bounded and is extremely sensitive to external parameters and initial values. Therefore, the chaos-based population initialization can traverse the search space within a certain range according to its own rules without repeating, so that the algorithm can significantly improve the accuracy and convergence speed of the algorithm. Here, the logistic mapping equation is used for population initialization, and its expression is as follows:

(14) $$\begin{array}{c} cx_{n+1}=\mu cx_{n}\left(1-cx_{n}\right), \end{array}$$

where the parameters *μ*∈(0, 4] and *cx*_*n*_ ∈(0, 1); the larger *μ* is, the higher the chaos is. When *μ* = 4, the system is completely in a chaotic state.

(15) $$\begin{array}{c} x\left(i,j\right)=x_{\min}+r\text{and }\left(i,j\right)\times \left(x_{\max}-x_{\min}\right). \end{array}$$

The basic principle of chaotic initialization population is as follows: First, given an initial value of *cx*, the chaotic variables needed for initialization are generated through the logistic mapping equation (see (14)). Then chaotic variables are used to replace the random numbers in the standard initialization equation, that is, *r* and (*i*, *j*) in (19), until each dimension of all dragonfly individuals is traversed.

#### 4.2.2. Reverse Learning Strategy

Reverse learning is an optimized learning strategy proposed by Tizhoosh in 2005. At the same time, according to the probability theorem, it is proved that each randomly generated candidate solution has a 50% probability of being closer to the optimal solution than its reverse solution. The main idea of applying the reverse learning strategy in this paper is to set a reverse probability *p* in the iterative optimization process of the DA. After each iteration of the dragonfly population update, a random number *r*_*3*_ from 0 to 1 is generated. If *r*_*3*_ ＞ *p*, then combine the reverse learning strategy to optimize the population. In the search space, the reverse individual is generated from the current individual, and the better individual is selected from the two to enter the next generation, thereby attracting the population to approach the optimal individual and increasing the randomness while reducing the complexity of the algorithm. The formula is as follows:

(16) $$\begin{array}{c} x_{ij}^{*}=k\left(a_{j}+b_{j}\right)-x_{ij}, \end{array}$$

where parameter *x*_*ij*_^*∗*^ is the reverse solution of the *i*-th dragonfly in the population in the *j*-th dimension. Parameters *a*_*j*_ and *b*_*j*_ are the minimum and maximum values of the *j*-th dimension, respectively, and parameter *k* determines the reverse learning type.

The time complexity indirectly reflects the length of time in which the algorithm is executed. In the DA, it is assumed that the execution time required to initialize the parameters (under the condition that the population size is *N* and the spatial dimension is *n*) is *x*_*1*_, and the time to generate a uniform distribution is *x*_*2*_. The time required to find the fitness value is *f*(*n*); then the time complexity of the initial stage of the DA is as follows:

(17) $$\begin{array}{c} O\left(x_{1}+N\left(nx_{2}+f\left(n\right)\right)\right)=O\left(n+f\left(n\right)\right). \end{array}$$

Assuming that the execution time required for the iterative update of each dimension of the individual is the same, which is *x*_*3*_; the time for comparing the advantages and disadvantages and selecting the best after iteration is *x*_*4*_. Then the time complexity of the algorithm at this stage is

(18) $$\begin{array}{c} O\left(N\left(nx_{3}+f\left(n\right)\right)+x_{4}\right)=O\left(n+f\left(n\right)\right). \end{array}$$

Therefore, the total time complexity of the IDA is

(19) $$\begin{array}{c} T\left(n\right)=O\left(n+f\left(n\right)\right)+O\left(n+f\left(n\right)\right)=O\left(n+f\left(n\right)\right). \end{array}$$

In summary, the improved DA does not increase the time complexity of the algorithm solution compared to the DA.

The chaotic initialization strategy can improve the quality of the initial dragonfly population and the randomness of population distribution, and the reverse learning strategy can increase the diversity of the dragonfly population. By comparing and selecting individuals with better fitness, the algorithm's optimization ability can be enhanced, and the population evolution speed and the algorithm's operating efficiency can be improved. The process is shown in Figure 1.

The basic steps of the improved dragonfly algorithm (IDA) are as follows.

**Step 1 .**

The randomly generated population size is the initial population of *m*, and the position of each particle is initialized chaotically using equations (19) and (20), and the parameters required for the algorithm execution are set in advance.

**Step 2 .**

Calculate the fitness value *f*(*i*) of each dragonfly, from which the position of the optimal individual is defined as the position of the food source, and its fitness value is *f*_*food*_. The location of the worst individual selected is defined as the location of the natural enemy, and its fitness value is *f*_*enemy*_.

**Step 3 .**

Update the parameters, including the search radius *r*, the inertia weight *w*, the separation weight *s*, the alignment weight *α*, the cohesion weight *c*, the food attraction weight *f*, and the natural enemy dispersal weight *e*.

**Step 4 .**

Calculate the step vector, and update the position of the dragonfly according to equation (12) when there is a nearby dragonfly. When there is no nearby dragonfly, update the position of the dragonfly according to formula (13), and limit it to the maximum range [0, *L* − 1].

**Step 5 .**

Substitute the updated position of each dragonfly into the fitness function to obtain a new fitness value *f*(*i* + 1).

**Step 6 .**

If *rand* > *p*, perform the reverse learning operation according to formula (16), and select the individual who enters the next generation from the current individual and the reverse individual.

**Step 7 .**

Compare the fitness value of the individual with the optimal value *f*_*food*_ and the worst value *f*_*enemy*_. If it is better than *f*_*food*_, update the position of the food, and if it is worse than *f*_*enemy*_, update the position of the natural enemy.

**Step 8 .**

Determine whether the conditions for terminating the iteration are met; if they are met, exit the loop; otherwise, go to Step 3.

## 5. Application of Improved Dragonfly Algorithm for MWSNs

The mobile Sink path optimization problem is to find the shortest moving path, so that the mobile Sink can ensure the minimum energy consumption and path optimization and high reliability data collection in the monitoring area, which is a combinatorial optimization problem. Converting the mobile path planning problem of mobile Sinks into the classic traveling salesman problem, this paper proposes a data collection method for mobile sensor networks based on the improved dragonfly algorithm, which improves the efficiency and reliability of data collection, prolongs network life, and reduces network energy consumption. The corresponding relationship between mobile Sink path planning strategy and dragonfly predation behavior is shown in Table 1.

The IDA proposed in this paper carries out research on path planning of mobile Sink data collection in the data collection process of mobile wireless sensor networks. The data collection is mainly divided into 4 steps, which are described in detail as follows:

1. For the sensor nodes in the monitoring area, their networking adopts the classic LEACH hierarchical clustering algorithm, and the cluster heads are selected according to the node's communication capacity and remaining energy. When the cluster head selection is completed, the cluster head only has the node data information (node position, number of cluster member nodes, and corresponding remaining energy) in the area where it is located. The information between the cluster heads needs to be exchanged between the cluster heads to obtain the information of the entire network. At the same time, the cluster head node accepts data collection tasks.
2. Divide the monitoring network area. After data exchange between cluster heads, each cluster head saves the information of its surrounding cluster head nodes. By calculating the total cost of communication with the surrounding cluster head nodes and calculating the communication distance and communication energy consumption under the constraints of energy consumption and shortest moving path, the network is partitioned according to the size of the communication cost, and finally a staying position is determined in each clustering area to ensure the energy consumption balance of data collection.
3. Move Sink to determine where to stay in each monitoring area. Whenever the mobile Sink reaches a place in the monitoring interval, it will broadcast information to the surrounding area. After receiving the information, the cluster head sends the information summarized in the cluster to the mobile Sink, and the mobile Sink stores and records the collected information and serves for the next round of data collection.
4. Optimization of the movement path of the mobile Sink. The Sink node determines its own stay point based on the cluster head data information collected previously (cluster head residual energy and position coordinate information). After that, the improved dragonfly optimization algorithm proposed in this paper is used to optimize the moving path, which mainly includes initial value coding, position update, calculated fitness value, and the best decision update. The swarm intelligence algorithm dragonfly optimization algorithm does not need high requirements for the initial position of the mobile Sink, and the calculation is relatively simple, so that the mobile Sink data collection is maximized, energy consumption is minimized, and the network runs with high reliability.

In the dragonfly optimization algorithm, its focus is the calculation of the fitness function, and the position of each individual dragonfly represents a solution of the optimization function. The size of the food that the dragonfly individual finds depends on the optimization function. The better the function value, the better the position. With the iteration of the algorithm, the dragonfly individual will continue to approach the dragonfly individual with a better position than its own. In the end, most dragonfly individuals will gather near the optimal position, that is, find the optimal solution. The flow chart of the improved dragonfly optimization algorithm in the mobile Sink path planning work is shown in Figure 2.

Algorithm 1 shows the implementation steps of the path planning strategy of WSNs based on the improved dragonfly optimization algorithm (IDA).

## 6. Experimental Simulation Comparison and Analysis

In this paper, Matlab simulation software is used to study the mobile Sink path optimization problem of the wireless sensor network of the perception layer of the Internet of Things proposed by us. The experimental environment of the algorithm is 64-bit Windows 10, with 3.2 GHz processor and 32 GB memory, and the programming environment is MATLAB 2016b. In order to objectively compare the comprehensive performance of the IDA and those of the other three algorithms, the influence of the randomness of the algorithm on the experimental results is fully considered. The settings of the dragonfly algorithm are as follows: the number of populations *n* = 30, and the maximum number of iterations is 100. The parameters of the search radius *r*, the inertia weight *w*, the separation weight *s*, the alignment weight *α*, the cohesion weight *c*, and the food attraction weight *f* are all set to linearly decreasing weights, and the value range is [0.3, 0.9]. Assume that the mobile wireless sensor network nodes are randomly and evenly distributed in a two-dimensional space of 500 × 500 m^2^, and the scale of sensor nodes is 200. The number of simulation polls is set to 500. In each simulation, the sensor node has 10 data packets transmitted from the source node to the Sink, and each data packet has a capacity of 4 kb. The initial energy of the Sink is set to 50 J, the Sink moves in a uniform straight line at a speed of 5 m/s, and the initial energy of a common node is 1 J. The parameter settings of the mobile wireless sensor network are shown in Table 2.

In order to better illustrate the superiority of the proposed algorithm, this paper compares four data collection algorithms: random walking, artificial bee colony (ABC) algorithm [37], dragonfly algorithm (DA), and the improved dragonfly algorithm (IDA) proposed in this paper.

The mobile Sink patrols the cluster head nodes in the area to collect data. Movement path planning reflects the path length of the mobile Sink. The longer the length, the longer the collection time and the greater the energy consumed. Therefore, the shorter the path length of the mobile Sink, the better the network performance. The comparison of the path length of the mobile Sink of the four algorithms is shown in Figures 3 and 4.

The four simulation diagrams in Figure 3 show the moving path planning diagrams of the random walking method, artificial bee colony (ABC) algorithm, dragonfly algorithm (DA), and the IDA proposed in this paper. It can be seen from the four simulation diagrams that the random walking method has the longest moving path and is also chaotic. The artificial bee colony algorithm has a relatively good moving path, and it only has a small amount of partial path planning that is not very good. The basic dragonfly algorithm has poor path planning. The improved dragonfly optimization algorithm proposed in this article has the best path planning and the shortest and optimal moving path, which is also the most reasonable.

### 6.1. Average Network Energy Consumption

The average energy consumption of the network reflects the energy consumption of the wireless sensor network. It is an important manifestation of network performance indicators and most intuitively reflects the working life of the network. The network average energy consumption comparison of the four algorithms is shown in Figure 5.

It can be seen from the trend of the four network average energy consumption distribution graphs in Figure 5 that, with the increase in the number of network polls, the average network energy consumption of the four algorithms is gradually increasing, but their growth rates are not the same. It can be clearly seen that the increase of the energy consumption in the random walk method is the largest compared to the other three intelligent optimization algorithms. The network energy consumption of the three intelligently optimized algorithms is not much different. At the same time, from the comparison of the three optimization algorithms, the improved dragonfly optimization algorithm proposed in this paper has the lowest energy consumption and the smallest increase.

### 6.2. Three-Dimensional Energy Consumption Comparison

In order to more intuitively and effectively reflect the comparison of the network energy consumption of the four different data collection methods, we give a comparison of the three-dimensional network energy consumption of the four different data collection methods. In the three-dimensional graph, the horizontal axis and the vertical axis are the number of sensor nodes, and the *z*-axis is the network energy consumption of sensor nodes. The three-dimensional network energy consumption comparison of the four data collection methods is shown in Figure 6.

From the comparison of the three-dimensional energy consumption of the four algorithms in Figure 6, the network three-dimensional energy consumption of the random walk data collection method is the largest. The maximum energy consumption of its sensor nodes has reached 1 J, and the average energy consumption of sensor nodes is also between 0.6 J and 0.8 J, which is the largest energy consumption. The network energy consumption of the artificial bee colony algorithm and the basic dragonfly optimization algorithm is not much different, and their energy consumption is between 0.4 J and 0.6 J. The improved dragonfly optimization algorithm proposed in this paper has the lowest network energy consumption. The maximum network energy consumption is also around 0.4 J. In most cases, the average energy consumption of its network is between 0.2 J and 0.3 J. It can be seen that the network energy consumption of the improved dragonfly optimization algorithm proposed in this paper is the smallest.

### 6.3. Load Balance Comparison

Network load balancing is an important indicator of wireless network energy consumption and network life. The better the load balancing performance of the network, the longer the lifetime of the network. The load balancing of WSNs is generally expressed by load balancing factor (*L*_*LBF*_). *L*_*LBF*_ is defined as the reciprocal of the variance of all sensor nodes in the monitoring area. For example, the larger the *L*_*LBF*_ value, the better the network load balance. The specific calculation is as follows:

(20) $$\begin{array}{c} L_{LBF}=\frac{M_{c}}{\sum_{i=1}^{n_{c}}{\left(x_{i}-m\right)}^{2}}. \end{array}$$

In formula (20), parameter *M*_*c*_ is the number of sensor nodes. Parameter *x*_*i*_ is the number of sensing nodes in the *i*-th cluster head member. Parameter *m* is the average number of nodes of all cluster head nodes. The network load balance comparison of the four algorithms is shown in Figure 7.

It can be seen from the network load balance comparison graph in Figure 7 that the random walk data collection method has a large fluctuation in network load balance and is not balanced. The network load balance of the remaining three algorithms is not much different. But, from the perspective of the overall network load balance of the four algorithms, this paper proposes improving the dragonfly optimization algorithm to have a stronger network load balance performance.

### 6.4. Comparison of Network Latency

The network latency measures the real-time performance of different data collection methods by the transmission time of successfully received data packets. A piece of data is recorded as *L*_*s*_ at the sending time of the source node and *L*_*r*_ at the receiving time of the Sink node. Then the average transmission delay formula is

(21) $$\begin{array}{c} T_{\text{trans}}=\frac{1}{N_{s}}\sum_{i=1}^{N_{s}}\left(L_{ri}-L_{si}\right), \end{array}$$

where parameter *N*_*s*_ is the total number of successfully received packets. The network delay of the three algorithms is shown in Figure 8.

From the comparison of the network transmission delay of the four algorithms in Figure 8, it can be seen that, at the beginning of the algorithm simulation, the random walk method has the largest data transmission delay, and the initial transmission delay simulation reaches 3.5 seconds. The data transmission delay of the other three kinds of intelligent optimization algorithms is longer. This is mainly because the algorithm performs a series of calculations in the process of finding the optimal path. On the whole, as the simulation of the algorithm progresses, the improved dragonfly optimization algorithm proposed in this paper has a smaller transmission delay compared to the other three methods.

### 6.5. Comparison of Network Connectivity

Network connectivity generally uses continuous motion discretization to calculate network connectivity. That is, in a relatively short period of time, it is considered that the topology of the network does not change, and the network structure remains unchanged. For a network at a certain moment, the calculation of the connectivity rate of WSNs is generally determined by the perceptual node traversal method. Suppose that a sensor node is used as a reference, and the nodes connected to its one hop, two hops, and three hops are sequentially searched until the number of nodes connected to the initial sensor node no longer increases. The mathematical calculation formula of the network connectivity rate *C*_*con*_ is

(22) $$\begin{array}{c} C_{\text{con}}=\frac{N_{l}}{n}, \end{array}$$

where parameter *N*_*l*_ is the number of adjacent nodes within the communication range of the node parameter *n* is the number of all the sensor nodes in the entire network. The comparison of the network connectivity of the four algorithms is shown in Figure 9.

From the comparison of the network connectivity of the four algorithms in Figure 9, the network connectivity fluctuation range of random walking is the largest, and the network connectivity decline is also the largest. There is little difference in network connectivity between artificial bee colony algorithm and basic dragonfly optimization algorithm. The improved dragonfly optimization algorithm proposed in this paper has better network connectivity compared to the other three algorithms and has the smallest fluctuation range. Taking the time of 40 polling times as an example, the network connectivity of random walking is 0.42, the network connectivity of the ABC algorithm is 0.57, the network connectivity of the DA is 0.69, and the network connectivity of the improved DA is 0.76. The algorithm proposed in this paper has better network connectivity compared to the other three algorithms.

### 6.6. Comparison of Network Reliability

The reliability of the network *R*_*net*_ is composed of the sensor node connectivity reliability *I*_*1*_, network connectivity rate *I*_*2*_, and the network capacity *I*_*3*_ [37]. Its mathematical calculation formula is

(23) $$\begin{array}{c} R_{\text{net}}=0.2I_{1}+0.5I_{2}\\ =0.3I_{3}. \end{array}$$

The connectivity reliability of network nodes *I*_*1*_ refers to the reliability of end-to-end node connectivity. Generally, the reliability matrix is calculated based on the distance between WSNs sensing nodes. According to Monte Carlo analysis, the average node connectivity reliability value after 50 rounds is obtained. Parameter *I*_*2*_ is the network connectivity rate calculated by formula (23). The network capacity *I*_*3*_ is the network survival probability, which generally represents the ratio of the current network node survival nodes to the number of all nodes [38]. The comparison of the network reliability of the four algorithms is shown in Figure 10.

The reliability of the network is mainly composed of three parts, so its reliability influence parameters are relatively large. However, its trend is not much different from the change trend of network connectivity. The main reason here is that the network connectivity influence factor accounts for the largest proportion. From the comparison of network reliability in Figure 10, the network reliability of the random walking method is relatively the worst, in addition to the lowest car-building connectivity performance. In artificial bee colony algorithm, the network reliability is relatively poor. The network reliability of the basic dragonfly optimization algorithm is better. This paper proposes that the network reliability of the improved dragonfly optimization algorithm is better compared to the other three methods. This mainly depends on its path planning, the optimal transmission time is the shortest, and the network connectivity is the best.

## 7. Conclusions

Mobile wireless sensor networks are currently a hot research field for WSNs, and there are still many key issues that need to be solved urgently. Among them, this paper studies the data collection problem based on the path optimization of the mobile Sink as one of the hot research problems, and it is also one of the key technologies of the mobile wireless sensor network. This article addresses the problems of limited node energy, unbalanced energy consumption, unreliability, and long delay in the data collection process of mobile wireless sensor networks. A new mobile Sink path optimization mechanism based on the improved dragonfly algorithm to optimize mobile wireless sensor networks is proposed. Experimental simulation results show that the data collection strategy designed in this paper can improve the collection efficiency of mobile collection nodes, reduce the energy consumption of static sensor nodes due to the data of other static sensor nodes, and effectively improve the maximum survival time of wireless sensor networks. Overall, the algorithm proposed in this paper ensures network connectivity, improves network communication efficiency, balances node energy consumption, solves fault tolerance during transmission, satisfies network service quality, and improves the reliability of the network.

Although the research in this paper has improved the performance of the network, the computational complexity of the network is relatively high, and the transmission delay of the network is still relatively large. The next work is how to reduce the computational complexity of the network and further reduce the transmission delay of the network. The model established in the article is based on the assumption that the nodes are distributed on a two-dimensional plane, but, in practical applications, the layout of some wireless sensor networks cannot be simply regarded as a two-dimensional plane. In addition, the communication load borne by each static sensor node is different, and the importance in the network is also different. In the process of data collection, emphasis should be placed on reducing the communication pressure of static sensor nodes with a large communication load. There are other ways to improve the algorithm for solving this problem, and further research on these problems will be carried out in the future.

## Figures and Tables

**Figure 1:** The flow chart of improved dragonfly algorithm.

**Figure 2:** The workflow of path planning of mobile Sink with improved dragonfly algorithm.

**Figure 3:** Path planning comparison of mobile Sink (200). (a) Random walk. (b) ABC. (c) DA. (d) IDA.

**Figure 4:** Path planning comparison of mobile Sink (300). (a) Random walk. (b) ABC. (c) DA. (d) IDA.

**Figure 5:** Comparison of average network energy consumption.

**Figure 6:** Comparison of three-dimensional network energy consumption. (a) Random walk. (b) ABC. (c) DA. (d) IDA.

**Figure 7:** Comparison of network load balance.

**Figure 8:** Comparison of network latency.

**Figure 9:** Comparison of network connectivity.

**Figure 10:** Comparison of network reliability.

**Algorithm 1:** Pseudocode of path planning of mobile Sink with the IDA.

**Table 1:** The corresponding relationship between mobile Sink path planning strategy and dragonfly predation behavior.

Predation behavior of dragonfly	Path planning for mobile Sink
Dragonfly position	Position of all cluster heads
Food yield	Path length, data collection volume, energy consumption
Speed of looking for food	Data collection speed of mobile Sink
Food location with the highest yield	Shortest collection path of mobile Sink
Time required to prey on food	Time-consuming algorithm simulation

**Table 2:** Simulation environment parameter setting.

Parameter	Value
Network range	500 × 500 m^2^
Number of nodes	200
Communication radius	50 m
*V*_*Sink*_	5 m/s
Initial energy	1 J
*E*_*elec*_	50 nJ/bit
*E*_*fs*_	10 pJ/bit/m^2^
*E*_*mp*_	0.0013 vpJ/bit/m^4^
*l*	4000 bits
*d*_*0*_	$\sqrt{E_{fs}/E_{mp}}=87\text{ m}$

## Data Availability

The data used to support the findings of this study are available from the corresponding author upon request.
